# A Systematic Analysis on COVID-19 Patients in Inner Mongolia Based on Dynamic Monitoring

**DOI:** 10.1155/2021/5559187

**Published:** 2021-04-20

**Authors:** Lan Yu, Tianbao Li, Li Gao, Bo Wang, Jun Chai, Xiaoli Shi, Rina Su, Geng Tian, Jialiang Yang, Dejun Sun

**Affiliations:** ^1^Clinical Medical Research Center/Inner Mongolia Key Laboratory of Gene Regulation of the Metabolic Diseases, Inner Mongolia People's Hospital, Hohhot, Inner Mongolia, China; ^2^Geneis (Beijing) Co., Ltd., Beijing, China; ^3^Qingdao Geneis Institute of Big Data Mining and Precision Medicine, Qingdao, China; ^4^Department of Pulmonary and Critical Care Medicine/Key Laboratory of National Health Commission for the Diagnosis & Treatment of COPD, Inner Mongolia People's Hospital, Hohhot, Inner Mongolia, China; ^5^Medical Imaging Department, Inner Mongolia People's Hospital, Hohhot, Inner Mongolia, China; ^6^Telemedicine Center, Inner Mongolia People's Hospital, Hohhot, Inner Mongolia, China

## Abstract

COVID-19 has spread globally with over 90,000,000 incidences and 1,930,000 deaths by Jan 11, 2021, which poses a big threat to public health. It is urgent to distinguish COVID-19 from common pneumonia. In this study, we reported multiple clinical feature analyses on COVID-19 in Inner Mongolia for the first time. We dynamically monitored multiple clinical features of all 75 confirmed COVID-19 patients, 219 pneumonia patients, and 68 matched healthy people in Inner Mongolia. Then, we studied the association between COVID-19 and clinical characteristics, based on which to construct a novel logistic regression model for predicting COVID-19. As a result, among the tested clinical characteristics, WBC, hemoglobin, C-reactive protein (CRP), ALT, and Cr were significantly different between COVID-19 patients and patients in other groups. The area under the curve (AUC) of the receiver operating characteristic (ROC) curve was 0.869 for the logistic regression model using multiple factors associated with COVID-19. Furthermore, the CRP reaction showed five different time-series patterns with one-peak and double-peak modes. In conclusion, our study identified a few clinical characteristics significantly different between COVID-19 patients and others in Inner Mongolia. The features can be used to establish a reliable logistic regression model for predicting COVID-19.

## 1. Introduction

Since early 2020, there has been an outbreak of a novel highly infectious disease called coronavirus disease 2019 (COVID-19), which quickly spread globally. As reported by the World Health Organization (WHO), there are more than 90 million confirmed COVID-19 cases and 1.9 million deaths across 212 countries by Jan 11, 2021, and these two numbers are still increasing. COVID-19 is a new type of pneumonia with several kinds of clinical manifestations caused by severe acute respiratory syndrome coronavirus (SARS-CoV-2) [1]. SARS-CoV-2 belongs to the coronavirus family, whose members also cause infectious diseases like severe respiratory to viral cold, severe acute respiratory syndrome (SARS), and Middle East respiratory syndrome (MERS) [2]. By binding to angiotensin-converting enzyme-2 (ACE-2), SARS-CoV-2 primarily targets respiratory epithelium cells, which results in inflammatory response and thereby induces epithelium cell apoptosis. The transmission modes of COVID-19 are similar to those of SARS, including contact, droplet, airborne, vomit, fecal-oral, bloodborne, mother-to-child, and animal-to-human transmission [3, 4]. Based on the Diagnosis and Treatment for COVID-19 (Trial version 7) published on Aug 19, 2020, a suspected case is classified as a confirmed case if it has one of the following etiological or serological evidence: RT-PCR detection of SARS-CoV-2 nucleic acid is positive; viral gene sequence is highly homologous with known SARS-CoV-2; the SARS-CoV-2-specific IgM antibody and IgG antibody are positive; the SARS-CoV-2-specific IgG antibody turns from negative to positive, or the IgG antibody titer in the recovery phase is at least 4 times higher than that in the acute phase [5].

Similar to SARS, pulmonary dysfunction and fibrosis are the primary cause for the death of COVID-19 patients [6]. Cardiac arrest and total organ failure are the secondary cause, indicating that the immune system also participates in the course of disease progression [7–9]. The illness severity can range from mild to critical in the cohort, including mild (mild symptoms and no manifestations of pneumonia on imaging), moderate (fever, respiratory symptoms, and manifestations of pneumonia on imaging), severe (dyspnea, hypoxia, ≥30 breaths per minutes, and oxygen saturation ≤ 93% at rest, or more than 50% lung involvement on imaging), and critical (respiratory failure, mechanical ventilation required, shock, or multiorgan system dysfunction) [5, 10, 11]. Furthermore, some patients died from “consequent cytokine storm” due to total organ failure by viral inflammatory response [12, 13]. When plenty of cytokines release to blood circulation, they lead to electrolyte imbalance, metabolic acidosis, multiple organ dysfunction, and total organ failure. Therefore, it is critical to have early diagnosis and frequent monitor especially for patients with underlying diseases, whose immune systems could be suppressed and are sensitive to cytokine release.

Though the RT-PCR test is served as the gold standard technique to confirm the infection of SARS-CoV-2, the technique is time consuming and subject to false negative [11]. Therefore, other auxiliary tests combining clinical, molecular, and radiological features would be beneficial for diagnosis. In clinical, COVID-19 is mostly characterized by inflammatory exudative pulmonary lesions with symptoms including fever, dry cough, headache, myalgia, breathlessness, and asthenia [14, 15]. Although clinical tests are essential for diagnosis, the symptoms of patients at the early stage of COVID-19 could not be differentiated from common viral pneumonia. Thus, it is critical to study the association between cellular or molecular markers and the severity and prognosis of COVID-19. Recently, several strongly associated biomarkers, such as the lymphopenia (defined as lymphocyte count < 1000), elevated C-reactive protein (CRP), and lactate dehydrogenase (LDH), were identified [16, 17]. In addition, non- or less-specific myocardial biomarkers, such as creatine kinase (CK), elevated level of hepatic enzyme, d-dimers, interleukin-6, C-reactive protein, and procalcitonin, were also suggested to associate with the poor prognosis of COVID-19 [18–20].

It has been reported that clinical, molecular, and radiological features of COVID-19 patients are all varied with time. However, the dynamic patterns of COVID-19 patients have not been fully studied. For example, a series of clinical factors such as white blood cell (WBC), C-reactive protein (CRP), and lymphocyte (LYM) have been reported to be associated with COVID-19 progression in previous studies [21]. Dynamic monitoring of these inflammatory factors would be a benefit for developing a suitable plan as well as predicting disease outcome. COVID-19 is an acute infectious disease, and the early symptom is similar to common cold; however, some patients will develop rapid disease progression and multiple organ failures within only a few days from diagnosis.

Finally, previous studies have suggested that patients of different races or in different regions may have differences in COVID-19 progression, symptoms, and prognosis. Several studies have reported people living at multiple regions, such as Asia, Europe, and North America, presented different clinical symptoms of the disease. To date, about eighty thousand COVID-19 confirmed cases have been reported in China, worse more, there are nearly 31,021,218 confirmed cases with approximately 960 thousand deaths globally, and the number is more likely to increase [22]. Currently, most cases were from the United States, which accounts for nearly 80% of total cases globally. However, since the Inner Mongolia population has unique characteristics in terms of ethnicity, climate, and dietary culture, we conducted this study from multicenter hospitals across Inner Mongolia, aiming to investigate the difference among people living in Inner Mongolia, China, during the time of COVID-19 occurrence. We found several familial cluster cases which confirmed with the previous study indicting the possibility of human-to-human transmission of SARS-CoV-2 [23].

We conducted a retrospective cohort study from multiple medical centers in the Inner Mongolia autonomous region, China. This study is aiming to investigate the association between the clinical parameters and prognosis in Inner Mongolia, especially the time-series patterns. Moreover, we try to preliminarily study whether COVID-19 has the homogeneity across different ethnic groups, viral load, clinical features as well as transmission mode, and possible other influencing factors as well.

## 2. Materials and Methods

### 2.1. Cohort Population of the Study

This retrospective population-based cohort study was performed in eleven cities across the Inner Mongolia region of China. Seventy-five patients with COVID-19, 219 viral or bacterial acquired pneumonia patients, and 68 heath individuals of Han or Mongolian ethnicity were enrolled in the present study. All COVID-19 patients were laboratory-confirmed clinically diagnosed, and the admission date was ranged between January 21, 2020, and February 23, 2020. The criteria used for the diagnosis of COVID-19 was confirmed by RT-PCR as the following: RT-PCR detection of SARS-CoV-2 nucleic acid is positive, and viral gene sequence is highly homologous with known SARS-CoV-2. Pneumonia was classified combining with clinical features of fever and cough or cough phlegm and chest X-ray scanning, which show marked thickening of the lung texture and could hear moist rales or pronounced sputum purr in the lungs with stethoscope auscultation. Pneumonia patients and healthy people were randomly selected from hospitals within the last 6 months before the COVID-19 pandemic. The clinical information including age, gender, severity of disease, incubation time, and hospitalization with clinical lab exams at different points was collected. For COVID-19 and pneumonia patients, the clinical laboratory test results were collected from medical facilities for each patient on both the admission day to the hospital and monitoring during the entire hospital stay every two days. For healthy people, the clinical laboratory test results were collected on the date of regular health exam. Generally, lab exams were performed approximately every two days which included WBC, lymphocyte, neutrophils, hemoglobin, platelet, C-reactive protein (CRP), procalcitonin (PCT), alanine aminotransferase (ALT), aspartate aminotransferase (AST), lactate dehydrogenase (LDH), and serum concentration of creatinine (Cr). On admission day, patients were clinically diagnosed as mild-moderate, severe, or critical facilitating physicians to design the treatment plan according to the WHO classification for COVID-19 [5, 10]. Informed consent was waived since this retrospective study represents no more than minimal risk to subjects and will not adversely affect their rights.

### 2.2. Logistic Regression Model to Distinguish Patients with COVID-19 from Viral or Bacterial Acquired Pneumonia

Continuous variables were expressed as mean ± standard deviation, and categorical variables were presented as number of subjects (frequencies). The Wilcoxon rank-sum test was used for testing the difference of variables between COVID-19 groups and pneumonia or healthy people, respectively, with multiple correction tests, and the significance threshold was 0.05. A logistic regression model was built to distinguish COVID-19 from seasonal pneumonia identified by single or multiple laboratory features. Logistic regression was applied for the probability model for predicting the probability of an event by fitting a logic function/hypothesis function. The output of the logistic regression formula means the probability of *y* = 1 given *X* and *b*. *g*(*x*) is sigmoid function as the following:

(1) $$\begin{array}{c} P\left(y=1\;|\;X;b\right)=g\left(b^{T}\right)=g\left(b^{T}X\right)=\frac{1}{1+e^{-b^{T}X}}, \end{array}$$

where *b* stands for a linear coefficient of logistic regression, *X* stands for the features extracted from data, and *g*() stands for the function of sigmoid. In addition, this equation shown above predicts *P* as a function of *X*. Using this equation, note that as *bTX* approaches negative infinity, the result in the formula for *P* approaches zero, so *P* approaches zero. When *bTX* approaches positive infinity, *P* approaches one. Thus, the function is bounded by 0 and 1 which are the limits for *P*. Furthermore, the logistic regression model was used to predict the type of disease and receiver operating characteristic (ROC) curve was created for prediction model assessment and 95% confidence interval was calculated by Python package of statsmodels (v0.12.1).

## 3. Results

### 3.1. A Few Clinical Laboratory Features of COVID-19 Patients in Inner Mongolia Were Significantly Different with Those of Common Pneumonia and Healthy People

We reported a retrospective cohort study with 75 COVID-19 patients from multiple medical centers. All COVID-19 patients were confirmed by laboratory RT-PCR, along with randomly selected 39 patients with seasonal pneumonia, and 68 nonpneumonia healthy people (Table 1). The mean age of the four cohorts was 43.67, 36.12, 55.46, and 45.39, respectively, and the age of most COVID-19 patients was over 60. According to the WHO definition, there were 13 mild symptom cases, 48 moderate symptom cases, two severe cases, and one death which are due to COVID-19-related complication. The youngest COVID-19 patient was 17 months old with the diagnosis of mild, and a severe case of most aged patient was 86. The imported COVID-19 patient cohort includes 25 mild symptom cases and 25 moderate cases with 2 severity cases. Epidemiology investigation illustrated the average incubation period of COVID-19 was approximately 9 days and the longest incubation day was 26 days, which was consistent with previous studies [24]. The average hospitalization stay was 22 days. For epidemiology tracking, several patients had visited the city with COVID-19 patients and almost all confirmed cases were directly or indirectly related to other patients. In addition, the people participated in our study presented significant as family cluster and community-acquired transmission pattern (data not shown).

Almost all patients on admission day presented fever symptom, 16% with dyspnea, 28% with cough, 31% with fatigue, 64% with myalgia, 11% with diarrhea, and 21% with other atypical symptoms including abdominal discomfort, nausea/vomiting, and headache. The elderly and men have relatively high susceptibility to SARS-CoV-2, and previous studies also reported that MERS-CoV and SARS-CoV infected more men than female [21, 24]. One hypothesis is that women have relatively strong immune response ability including both innate and adaptive immune response, which might be due to additional X chromosome and sexual hormone [25, 26]. At admission, multiple lab exams were performed including white blood cell counts, lymphocyte, neutrophil granulocyte, hemoglobin, platelet count (PCT), C-reactive protein (CRP), and several hepatic enzymes. The comparison of serum creatinine (Cr), white blood cell count (WBC), CRP, neutrophil granulocyte, hemoglobin, and aspartate aminotransferase (AST) showed statistically significant difference between COVID-19 and seasonal pneumonia patients as well as nonpneumonia (Figure 1). The COVID-19 patients could be distinguished by the combination of clinical laboratory features, while no significant showed between seasonal pneumonia and nonpneumonia patients.

### 3.2. Logistic Regression Model on Clinical Laboratory Features Can Diagnose COVID-19 with Relative Good Performance

On the diagnosis of COVID-19, most patients presented with increasing lymphocytopenia and neutropenia; furthermore, most patients also had elevated ALT, lymphocyte, and creatinine. In order to evaluate the performance of the statistical model, we selected two cohorts (COVID patients and pneumonia patients) to find out whether the logistic regression model could separate those variables accurately. The results showed our logistic regression model could differentiate COVID patients from healthy people within three clinical laboratory features, which indicated our model has good performance (Figure 2(a)). Lymphocytes, white blood cells, and CRP associated with disease severity and prognosis were chosen to further evaluate the model performance. The cutoff value of 0.5 was applied in the model to evaluate the effect on the model, and the cutoff values of lymphocytes were 8.34, CRP was 98.60, and WBC was 9.17. The AUC of lymphocytes, CRP, and white blood cell were 0.68, 0.56, and 0.76, respectively, indicating lymphocytes and white blood cell were closely associated with the progression and prognosis of COVID-19 and were a good indicator for COVID-19 diagnosis. The AUC of all three features reached 0.82 with a 95% confidence interval of 0.856 to 0.909 and was relatively better than a single marker, which is approved that COVID-19 had multiple influencing factors and the result would assist health professionals to develop better diagnosis estimation for patients (Figure 2(b)).

### 3.3. There Are Several Dynamic Patterns of C-Reactive Protein in COVID-19 Patients in Inner Mongolia

In order to monitor the CRP which would reflect the disease severity, progress, and effectiveness of treatment, we plotted the dynamic monitoring figure. According to CRP result on the admission day, CRP values were collected as initial monitor point and continue to monitor every other day for several time points. As shown in Figure 3(a), there were five patterns during hospital stay, indicating the treatment efficacy. The CRP level of most patients had been decreased after 4 days and responds to treatment within a week (Figure 3(b)). Another specific pattern is shown in Figure 3(c).

Figure 3(b) shows the dynamic monitoring of CRP pattern from patients; the first peak was showing at the first week of hospital stay, which means patients' condition deteriorated for a period of time; they started to respond to treatment after hospital stay, showing that the treatment was effective and CRP level remained stable, still not fully recovered to normal though.

## 4. Discussion

Coronavirus is a family of enveloped single-stranded positive-sense RNA viruses and has a worldwide distribution. Six types of coronaviruses in the world can infect humans, and most infections are mild. However, severe acute respiratory syndrome (SARS-CoV) and Middle East respiratory syndrome (MERS-CoV) caused a large pandemic outbreak, and the mortality rate was approximately 10% and 30%, respectively [27]. Comparing with the SARS-CoV outbreak in 2003 which was a high-pathogenicity virus with high mortality, SARS-CoV-2 seems to be relatively more contagious with approximately 2% [28]. However, people infected with SARS-CoV-2 could develop neutralizing antibody and have prolonged disease progress. The fact might illustrate the following two phenomena: firstly, in addition to the respiratory system, SARS-CoV-2 might cause multiple organ damages, including gastroenterological, and neurological, kidney damages, and even total organ failure.

Similar to other coronaviruses, SARS-CoV-2 also utilizes an angiotensin-converting enzyme-2 (ACE-2) functional receptor which is widely expressed in vascular endothelial cells and renal tubular epithelium, hepatic cells, neuron, and pulmonary and gastrointestinal systems. There are several hypotheses trying to explore the underline mechanism of SARS-CoV-2 infection, development, and efforts to deliver effective treatment and vaccination. To date, the mechanisms of immunopathology of SARS-CoV-2 infection include both innate and adaptive immunity. The epithelium of the lungs serves as the physical barrier, and epithelial cells, dendritic cells, and macrophages can trigger proinflammatory response of macrophages in bronchoalveolar cells. Those cells serve as an initial immune defense against viruses. Previous studies indicated that the macrophage accumulation or depletion was associated with severity of disease [29]. Moreover, neutrophils play a critical role in acute inflammatory response of bronchoalveolar. Therefore, elevated neutrophils are believed to produce reactive oxygen species, which is considered as the potent antibacterial mechanism. In one situation, virus infection could directly infect lymphocytes resulting in cell apoptosis. Another situation is that it could also destroy the lymphocyte-produced organs, such as bone marrow or thymus, interfering lymphocyte production or dysfunction.

The early stage symptoms of COVID-19 include dry cough, fever, chill, tiredness, and upper respiratory symptom shortness or difficulty breathing, and some atypical symptoms, such as gastrointestinal discomfort, diarrhea, etc. [30, 31], which is consistent with the previous report of early stage of SARS and seasonal influenza [32, 33]. COVID-19 patients usually have decreased white blood cell count and lymphocyte cell count caused by suppressed immune response resulting in sequential infection. Though decreased lymphocyte count is not a specific factor for COVID patients, it can distinguish other common bacterial and viral infection, and it could only present in the late stage of the disease. CT imaging features of SARS-CoV-2 are highly sensitive for patients who have false-negative RT-PCR results. Moreover, CT image could be a good indicator for monitoring patient disease prognosis as well as therapy effectiveness. The typical features from the CT exam for SARS-CoV-2-infected patients are bilateral lung lobe involvements and ground-glass opacities (GGO) shown in the early stage of the disease, followed by pulmonary consolidation, increasing the area of GGO and fibrosis shown in late stage [34, 35]. Finally, the pulmonary tissue turned into “white lung” which leads to severe dyspnea requiring mechanical ventilation and results in septic shock, total multiple organ failure, and cardiac arrest due to increased viral titers.

In our study, the clinical laboratory test of CRP showed significant difference between COVID-19 patients and control. CRP, secreted by the hepatocytes, is a well-known indication of inflammation in the inertial thinking way [36, 37]. The elevated CRP is founded not only in the acute phase of inflammatory disease but also in most chronic coronary and metabolic diseases, such as cardiovascular disease, diabetes, and obesity [38]. However, another important role of CRP is to regulate the human innate immune process and adjust the interaction between the inflammatory intruder and the immune system. It is logical that among the COVID-19 cases, the level of CRP was increased as the disease was diagnosed. Furthermore, three types of dynamic elevation patterns were revealed in our study; the value of CRP was gradually risen at the beginning of the hospitalization in pattern 1, signifying that the immune response was activated. As the treatment progresses, the SARS-CoV-2 was eliminated, and the level of CRP decreased. The CRP in the patients of pattern 2 had not shown an obvious peak but a flattened one, probably because of the testing time. That is, the sample or hospitalization time point was later than the CRP increasing time; there is another probability: the SARS-CoV-2 load was not enough to induce a strong reaction of the host defense, and the virus was wiped out soon. As far as pattern 3 is concerned, 2 peaks were shown in sequential order. This phenomenon might be indicated that CRP played a pleiotropic role in the process. Either anti-inflammation or proinflammation could be the major role in the different phases of the disease. The first peak of CRP might be the anti-inflammation activation when SARS-CoV-2 infected the host at the beginning, while the function of the second peak of CRP might largely rely on the context, either the relapse of the SARS-CoV-2 eliciting the reactivation of the complement pathway or the change of complement components induced by CRP, leading to the proinflammation course. In summary, the CRP-activated complement pathway is different from the activation mediated by antigen-antibody complexes, with rarely activated late phase component proteins.

## 5. Conclusion

In this study, we collected clinical data from multicenter hospitals in Inner Mongolia, China. We performed statistical analysis of clinical laboratory features associated with SARS-CoV-2 infection between COVID-19 and common pneumonia patients. Second, we further explore the dynamic changes of clinical parameters during the incubation period as well as hospital stays. This study provides primary results to benefit health care physicians in diagnosis evaluation.

## Figures and Tables

**Figure 1:** Clinical characteristic comparison between COVID-19 among pneumonia and healthy people. ns presents no significant, “∗∗” presents *p* value < 0.01, “∗∗∗” presents *p* value < 0.001, and “∗∗∗∗” presents *p* value < 10-8 which has been added into the figure legend.

**Figure 2:** (a) Logistic regression model for COVD-19 prediction with single or multiple laboratory features and applied for probability model for predicting the probability of hypothesis function. (b) The area under the curve of receiver operating characteristic of different clinical markers associated with COVID-19 for leukomonocyte, CRP, and white blood cell, respectively.

**Figure 3:** Dynamic monitoring of C-reactive protein in COVID-19 patients. (a) Detected CRP pattern with dynamic monitoring. (b) CRP response in a specific pattern of individual patient.

**Table 1:** Patient cohort information.

Clinical variable	Category	COVID-19	Imported COVID-19	Pneumonia	Control
Age	Mean (range)	43.67 (1-86)	36.12 (25-27)	55.46 (1-95)	45.36 (1-89)

Gender	Male	38	25	126	40
	Female	37	27	93	28

Severity degree	Mild	13	25	95	—
	Moderate	48	25	128	—
	Serious and death	3	2	0	—

Incubation time	Average (days)	9.22 ± 5.83	—	—	—

Hospitalization	Average (days)	22.28 ± 7.55	17.42 ± 8.23	—	—

## Data Availability

The data used to support the findings of this study are available from the corresponding author upon request.
